This article has been retracted.

# Research on Real-Time Tracking Algorithm of E-Commerce Logistics Information Based on Blockchain Technology

**DOI:** 10.1155/2022/7006506

**Published:** 2022-09-16

**Authors:** Yanjie Zhu

**Affiliations:** School of Business, Xuchang University, Xuchang, Henan 461000, China

## Abstract

In order to solve the problem of distrust of a large number of nodes under the overly centralized and centralized information transfer mode, a research method of real-time tracking algorithm of e-commerce logistics information based on blockchain technology is proposed. The application background of blockchain technology in real-time tracking algorithm of e-commerce logistics information is firstly described. Also, the blockchain technology, logistics information real-time tracking algorithm, cryptography technology, blockchain consensus algorithm, blockchain application scenarios, and other related technologies are analyzed in detail. Then, the blockchain model of real-time tracking of e-commerce logistics information is established, and it is found that data will be stored on the chain only when more than 51% of the nodes in the distributed system confirm that the data are valid. Otherwise, the data on the chain cannot be affected. Finally, the model description and hypothesis of real-time tracking of e-commerce logistics information based on blockchain technology are verified to provide guarantee for improving real-time tracking of e-commerce logistics information.

## 1. Introduction

Blockchain technology is based on a decentralized distribution ledger database, which is a new distribution infrastructure and computing paradigm [1]. Digital cryptocurrencies and finance are among the earliest applications of blockchain technology. Blockchain was first used in the financial industry. In the financial industry, it can be further subdivided into three subfields. Bitcoin was the first breakthrough for the public to understand blockchain technology. The digital cryptocurrency blockchain is called the era of blockchain 1.0, the application of blockchain technology in the securities and financial industry is called the era of blockchain 2.0, and the application of blockchain technology in the natural layer can be called the era of blockchain 3.0, such as the logistics industry, power distribution industry, and the Internet of Things industry [2]. Blockchain technology follows the technology on the Internet. In the future, the development of a new generation of technology at the bottom of human beings will affect the industry, and the proportion of trade volume to GDP is still high. Currently, we are looking for new technologies to “reduce costs and increase efficiency” for the logistics industry. Therefore, learning blockchain technology in the logistics industry is an important theoretical and practical concept [3].

## 2. Research Background

In recent years, with the rapid development and wide application of new generation technology in China, all walks of life have realized their own development bottlenecks [4]. Under such a development background, enterprises rapidly change their development ideas, actively embrace the development trend of digital economy, and vigorously promote the digital construction of enterprises, to achieve the purpose of enterprise business transformation. The main goal of the enterprise digital transformation is to realize the intelligent upgrading of the enterprises through the comprehensive and systematic digital remodeling of the enterprises and to build the enterprise into a future-oriented smart enterprise. Also, the digital transformation is the main means and core path to build a smart enterprise. The continuous progress of technology and industrial development has gradually become an important fuel source and driving force to promote enterprise informatization in the new era [5]. Under the continuous promotion of epoch-making core technology of enterprise informatization in a batch of emerging fields such as artificial intelligence, Internet of Things, big data, and blockchain, the production and living mode of the society has undergone a qualitative change. Enterprise informatization implements agile manufacturing and integrated manufacturing with customer demand; in space, enterprise informatization brings together in virtual form, which greatly promotes the process of digitization and informatization of the society. The application of these new technologies has rapidly promoted the process of social informatization and digitization, greatly reduced the cost of production management, and improved the efficiency of social operation and development speed. With the gradual maturity of digital technologies such as the Internet of Things, big data, 5G, and blockchain, the digital and network characteristics of production are becoming more and more obvious. The rapid development of science and technology is repowering the assets, equipment, and organizations of enterprises. At present, the development of blockchain industry is in the 2.0 era and is evolving to the 3.0 era, but a large number of infrastructure construction, standard formulation, and technical problems still need to be implemented and solved. The characteristics of logistics industry with large volume and multiple and scattered participants are consistent with the decentralized and distributed processing characteristics of blockchain. Blockchain technology can speed up the “cost reduction and efficiency increase” of the whole logistics industry, promote the transformation and upgrading of the logistics industry, and improve the efficiency of the logistics industry [6].

## 3. Introduction of Blockchain Technology and the Related Technologies of E-Commerce Logistics Information Real-Time Tracking Algorithm

Essentially, blockchain technology is a fork of proof technology. The so-called data distribution is not at the location of the data server but is stored in various parts of the network. The network directly realizes data sharing, replication, storage, and synchronization. Regardless of the form of storage of data, the user needs the storage device. There are two main types of data storage devices: direct zone storage and network-based storage. Blockchain is the archive of blockchain technology. A blockchain consists of “blocks” that are linked together in time [7]. Each “block” contains the same information. Blockchain technology was first used in bitcoin. Each block lists the exchange party and exchange rate, the time (a string of fields that record the time), the hash value and the hash value of the previous block, and so on. Each block is connected to the corresponding hash value. Form a chain from timestamps [8]. If the blockchain is likened to a list, then a block is the page of the list, written to a file connection. Information placed on the distributed network is validated and de-identified. Once the file is uploaded and verified, it will not be affected [9]. Each block contains the following information shown in Table 1.

The block header is written into the “news page” of the block, including blockchain version number, hash value of the previous block, Merkle root, timestamp, hard target, nonce, and so on. Among them, the blockchain version number indicates the version [10]. The number is valid for it and the rules agree. The hash value of the previous block corresponds to the number of the previous block. Use Merkle base to quickly query the relationship and specify the time when the block was created [11]. The difficulty target is the number of zeros whose block hash value starts with a string of zeros in a blockchain; however, timestamps will never lie because the past parts of the blockchain cannot be modified in any way. In the blockchain, the timestamp is the part of the area that contains specific information, and the information it contains always exists. Nonce is the ultimate solution for assembling the BLOCK POW approval mechanism. It can be explained in the following “approval mechanism” that how to implement the approval mechanism of proof of work (POW) [12].

Blockchain technology mainly applies hashing and Merkle tree structures, which are hash binary trees, as a data representation used to quickly summarize and verify the integrity of complex and regular data [13]. This binary tree contains cryptographic hashes. Data types are used to declare variables, and the program assigns different sizes of space according to different data types during running. Each block in the blockchain contains all the transactions that occurred in that block and is represented as a Merkle tree. In the bitcoin network, Merkle trees are used to layer together the transaction records generated by a block [14]. To generate a healthy Merkle tree, it is necessary to recursively run the hash algorithm on the hash node to hash it and record the transaction records that are updated immediately into the Merkle tree until there is only one hash node left, which is the Merkle root. The Merkle root structure is shown in Figure 1.

Merkle trees grow from the bottom up [15]. As shown in the figure, the original data of L1, L2, L3, and L4 transactions are, respectively, at the bottom. After hashing, four hashes of 0-0, 0-1, 1-0, and 1-1 are generated, and every two of the four hashes are concatenated and hashed again to produce the hash of the next level. It is similar to the upper level hash, a higher-level hash generated by two hashes in series [16]. If there is an odd number of hashes that makes it impossible for a single hash to pair in concatenation, a hash is copied so that the hash of the whole level is even. Each level of hashing results in the highest-level hash value, which is called the Merkle root. HashQ is to transform an input of any length into a fixed length of hash output by a hash algorithm, which is the hash value. If you want to find and verify the authenticity of a transaction, you only need to get the corresponding hash value path [17]. In this way, it is possible to quickly verify whether a transaction exists in the blockchain. The current classification and advantages and disadvantages of blockchain are shown in Table 2.

The core of e-commerce logistics operation system is to collect and process data and information and give feedback to decision makers and management personnel, so as to facilitate enterprises to carry out reasonable coordination and control of goods circulation and reduce the cost of storage, scheduling, and transportation while ensuring the smooth flow of goods in all departments. Through logistics management innovation, reduce logistics costs and improve the quality of logistics service to enhance the market competitiveness of enterprises. The operation architecture of e-commerce logistics is shown in Figure 2.

Layered logistics information real-time tracking algorithm of blockchain is shown in Figure 3.

The external operation system of the blockchain logistics system is shown in Figure 4.

The external operation system of the blockchain logistics system is shown in Figure 5.

The external blockchain system can be subdivided into order system, logistics transportation system, and supply chain finance system according to the specific type of information transmitted [18, 19]. The internal blockchain logistics system can be subdivided into procurement management system, warehouse management system, production management system, and financial data management system according to the type of information transfer. The structure of blockchain logistics management system is shown in Figure 6.

E-commerce logistics transportation system should have enterprises to notify the logistics company to come to collect pieces, upload and share logistics information in real time through logistics companies, confirm the delivery through customers, and carry out other functions. When packaging a new block, logistics companies mark the corresponding logistics information with the customer's address [20, 21]. Customers can look up their tagged hash values in the blockchain and send the private key signature to the logistics company. Hash values are the immutable and determined core basis of the potential and the most important aspects of blockchain technology. It retains the authenticity of the data recorded and viewed and the integrity of the blockchain as a whole. As the query certificate, the logistics company will then send the logistics information corresponding to the hash value to the customer, and the customer can compare the logistics information with the hash value to confirm that the logistics information will not be tampered with. If they are the same, the logistics information can be backed up and stored for future use in case of disputes. From encryption to hash algorithm, two points are particularly important. The first point is that it is difficult to reverse derive the original data based on the hash value, and the second point is that the probability of a hash conflict is very small. After the customer confirms the receipt of the goods, the customer sends the receipt information signed by the private key to other nodes [22, 23]. The bank collects confirmation of receipt information within a certain period of time and packages it into a new block to add to the blockchain. When a block is successfully added to the blockchain, the transaction recorded in the new block is confirmed to have been completed. E-commerce logistics and transportation system is shown in Figure 7.

A new block chain decentralized authentication technology is formed by combining asymmetric encryption technology, P2P network, hash operation, and other basic technologies. Instead of innovating and creating the underlying technology, the technology combines many technologies. The bitcoin blockchain uses asymmetric encryption algorithms to authenticate corresponding accounts. Bitcoin users randomly select a private key and then generate the corresponding public key to be disclosed to other users in the blockchain. After certain hash operation, this public key is the bitcoin address of this user, and other users can transfer money to this user through this address. Because of asymmetric encryption, other nodes can use the public key to verify the identity of a user and whether the information is sent by the key owner. A third party acquiring a user's public key cannot reverse its private key, which ensures that the user's transfer information cannot be forged. Also, because the same key is used for both encryption and decryption, this key is not made public. The process by which a user marks information with a private key is also known as “digital signature.” The process of uploading and billing transaction information in blockchain is as follows:

(1) $$\begin{array}{c} \begin{array}{c} A\text{Trading Information}\overset{\text{private key}}{⟶}\text{encrypted information}\overset{\text{public key authentication}}{⟶}\text{Transaction Information Announcement}\overset{\text{Miner bookkeeping}}{⟶}\\ \text{add to blockchain}⟶\text{Transaction complete}. \end{array} \end{array}$$

One of the biggest features of blockchain technology is the use of distributed node network system. In blockchain, consensus mechanism is the core content. Blockchain is a storage system, and the storage system is even thinner. Blockchain is a distributed storage system with no administrator, and every node has all the data. In a blockchain network, all nodes need to follow the same rules, which is the consensus mechanism. Consensus mechanism plays a role in determining whether new blocks can be created in blockchain networks. Consensus mechanism is a rule that every node must follow. It is also one of the four core technologies of blockchain. The consensus mechanism mainly plays a role in coordinating all node accounts in the blockchain network. The data storage of each node depends on the end result produced by the consensus mechanism. Without consensus, blockchain systems cannot function properly. Consensus algorithm is used to implement consensus mechanism in distributed systems. In a blockchain system, the algorithm that reaches a consensus on the sequence of transactions in a time window is a consensus mechanism. The consensus mechanism determines the degree of trust between the nodes of the blockchain system and the degree of external trust in the data on the blockchain. There are many kinds of consensus algorithms, but there is no universally agreed algorithm at present, and each algorithm applies to different scenarios. Currently, consensus algorithms commonly used in blockchain can be roughly divided into algorithms based on BFT idea for solving Byzantine problems and CFT algorithm for solving common node errors. The basic process of CFT algorithm is similar to two-stage submission, in which multiple nodes first obtain the right to send data, and the successful node is sent to all nodes for confirmation to get the confirmation submission data of most nodes. In order to solve this problem, the article proposes how to keep the consensus of other generals under the condition that some generals are known to have been influenced by false information or mutiny. This problem is known as the Byzantine general problem. In the Byzantine consensus algorithm, the number of secure nodes *R* is larger than the number of insecure nodes *E*, and under ideal circumstances, *R* wants the voting result to be uniform. Therefore, the Byzantine consensus algorithm has the following two situations. (1) If party *E* gives up voting, the result cannot be affected, so the result can also be obtained when the total number of votes is *P* < *R*. (2) In the least ideal case, *R*/2 people agree and *R*/2 people oppose. In this case, *E* node can manipulate the result, so *P* > *R*/2 + E. So, there are the following inequalities:

(2) $$\begin{array}{c} P>\frac{R}{2}+E\text{,}\\ P<R\text{.} \end{array}$$

The following inequality can be obtained from the above inequality:

(3) $$\begin{array}{c} R>\left(\frac{R}{2}\right)+E\text{.} \end{array}$$

The following inequalities can be inferred from the above inequalities:

(4) $$\begin{array}{c} R+\left(\frac{R}{2}\right)>R+E\text{,}\\ \left(\frac{3}{2}\right)R>ALL\left(\text{total number of nodes}\right)\text{.} \end{array}$$

Therefore, the final inequality is

(5) $$\begin{array}{c} R>ALL\left(\frac{2}{3}\right)\text{.} \end{array}$$

## 4. Blockchain Application Scenarios

Blockchain application scenarios mainly include data storage and smart contracts. The emergence of blockchain technology provides an excellent solution to data security problems. Blockchain makes use of a network system composed of distributed nodes and adopts asymmetric encryption and hashing cryptographic algorithms to ensure data security and integrity. All distributed nodes in the blockchain will jointly maintain data to achieve multinode storage of data copies. Because there are enough nodes, in theory, unless all nodes are destroyed, the account will not be lost. The security and reliability of account data can be guaranteed. In distributed nodes, the overall operation is not affected when there is a node failure, and each node does not need to disclose its identity during data transmission to protect the privacy of the node. Blockchain uses consensus algorithms to solve the transmission problem of distributed data. Data will be stored on the chain only when more than 51% of the nodes in the distributed system confirm that the data are valid. Otherwise, the data on the chain cannot be affected. Smart contracts are logical codes developed by specific programming languages and run on a distributed network composed of blockchains. The execution of contracts is judged according to business states and driven by business events such as transactions. Disseminate and implement electronic contract agreements through information means. After all the business entities confirm the smart contract, the content of the contract is converted into executable code and then stored in the chain. The code encapsulates the business state, transformation rules, triggering conditions, and event response rules after triggering. The program code of a smart contract is executed by a specific virtual machine, and when triggered by a business condition, the calling code performs a response based on the state. The deployment and execution process of smart contract is shown in Figure 8.

## 5. Establishment of Real-Time Tracking Model of E-Commerce Logistics Information Based on Blockchain Technology

The logistics information traceability mechanism model based on blockchain technology is a decentralized distributed data storage technology. All data information will be stored in multiple nodes or all nodes to ensure the authenticity and transparency of transaction data, prevent transaction data from being tampered with, and establish a safe and centerless credit system. Offline nodes, including scattered logistics resources such as vehicles, yard stations, and goods sources, are combined with the model of no vehicle carrier. In essence, it is a derivative of the crowdsourcing mode in the logistics industry. The blockchain logistics information traceability mechanism is a point-to-point transmission network based on P2P technology. The communication between the two parties does not rely on the central control node, but two parties automatically generate transaction information. Then, they broadcast the transaction to the entire web. It effectively solves the problems of scattered resources and asymmetric information communication in the logistics industry and realizes the point-to-point transaction without relying on the centralized service provided by the intermediary platform. In addition, hash function, asymmetric encryption algorithm, and Merkle tree can ensure automatic, safe, and confidential online transmission of offline logistics information such as vehicles, stations, and sources of goods, providing efficiency and security guarantee for the information transmission of logistics information traceability platform based on blockchain technology.

The real-time tracking algorithm of logistics information based on blockchain is mainly divided into four parts: the application layer of reality consciousness, the consensus layer of core consciousness, the virtual consciousness network layer, and the basic consciousness data layer. The basic consciousness data layer contains specific block and chain structure, in which the block body encapsulates the specific transaction hash value, which represents the record of data information and transaction quantity in the process of logistics transaction. The virtual network consciousness layer is responsible for the dissemination, verification, and exchange of information in the blockchain system. In the logistics information traceability mechanism, the information exchange between various carriers and information service providers is realized through the point-to-point network technology. One-way contact between each other will not form any conflict. Point-to-point technology can also help some lost nodes to call the standby data stored by other nodes in the whole network during data download, so as to obtain faster download speed. The transmission mechanism of transaction information relies on broadcast between distributed nodes and point-to-point data transmission. The shipper releases the logistics demand on the logistics information blockchain, the transporter receives the goods, the transporter sends the goods, and the transporter delivers the goods to the consignee. The transaction process information, such as the receipt of goods after the consignee confirms that the goods are in good condition, will be transmitted through the transaction information transmission mechanism, and these kinds of information will be sealed in the block after hashing. Asymmetric encryption algorithm will encrypt the transmission of transaction information between each node on the logistics information traceability blockchain, including shippers, transporters, carriers, and consignees, to ensure the protection of transaction privacy between each other. The core consciousness consensus layer refers to sharing authorization consensus mechanism, in which the transportation provider, information service provider, and postal administration (supervision party) as the “board of directors” are responsible for voting and verifying the transaction behavior and data. If the board of directors passes the transaction, the corresponding block will be linked to the main chain and the transaction will continue to the next step. The generation of “board of directors” can realize the balance between the current social structure that cannot be completely decentralized and the concept of complete decentralization of blockchain. The “board of directors” is generated by the voting of the whole network nodes of blockchain and is responsible for verifying and passing the real-time generated blocks. The application layer of realistic awareness refers to the logistics information traceability architecture based on blockchain technology, aiming to solve the problems of insufficient process control and low information transparency in the logistics industry. The whole architecture is based on the form of alliance chain, and the information service provider (owner) and the postal administration (supervisor) have higher management authority to manage the whole system, mainly including computer data management and industry supervision and management. They also have veto power over transactions, and rules with absolute regulatory authority are automatically enforced through smart contracts to eliminate the need for individual will. Other distributed nodes under the framework of alliance chain include transporter, carrier, shipper, and consignee, in which each subject can change owner at any time. However, participants' credit records, transaction data, and other information will be encapsulated in individual blocks, so that when participants trace logistics information back to blockchain to participate in service activities again, the stakeholders verify the credit information of the transaction party and finally choose the satisfied participants as partners.

### 5.1. Blockchain Technology Architecture for Real-Time Tracking of E-Commerce Logistics Information

E-commerce logistics information real-time tracking blockchain technology architecture is composed of data layer, network layer, consensus layer, incentive mechanism layer, intelligent contract layer, and specific application layer, which contains a variety of blockchain underlying technology, such as logistics transaction record hash data block and asymmetric encryption algorithm (ECDSA). The network layer includes the logistics information transmission mechanism and the logistics information traceability blockchain access mechanism based on P2P network. The consensus layer adopts the consensus mechanism of stock authorization certificate. Integrate the acquisition and distribution of order income and the incentive mechanism of information service providers for transportation providers into the blockchain system. Its content mainly includes value creation, distribution mechanism, and profit model of blockchain. The contract layer mainly includes various scripts, smart contracts, and programmable computer languages, in which the contract information occurring on the logistics information traceability blockchain will be automatically signed in the form of smart contracts, and the parties agree that the contract will be automatically performed after the content of the agreement is realized. Smart contracts are implemented using hash algorithm, go language, and asymmetric encryption algorithm. The contract between the carrier and the information service provider can be signed in the computer credit environment. The application layer represents the application cases of blockchain in logistics, medical treatment, intellectual property, and other industries. In this traceability mechanism, the chain mechanism with timestamp, the revenue distribution mode of logistics information traceability blockchain, and the distributed consensus mechanism between nodes are the most innovative features of blockchain technology.

The technical architecture of blockchain for real-time tracking of e-commerce logistics information is shown in Figure 9.

The data layer of real-time tracking e-commerce logistics data blockchain usually includes narrow chain, data block structure, and chain structure. Narrow blockchain is a data storage ledger that synchronizes each node in a decentralized logistics information traceability system. Data block structure refers to logistics information block, which is a container data structure containing logistics transaction information. Chain structure refers to the main chain formed by linking the current block that has been verified by the dpos consensus algorithm to the previous block. The blockchain structure of real-time tracking of e-commerce logistics information is shown in Figure 10.

In e-commerce logistics information real-time tracking blockchain, smart contract is a tool for all distributed nodes to reach agreement. The contract contains the terms of rights and obligations of the information service provider, the carrier, the shipper and the consignee, the time and date of fulfillment of the commitment, the punishment regulations, and the electronic signatures of all parties. When the conditions on the contract are met, the smart contract automatically performs the next task. When the conditions specified in the contract cannot be fulfilled, the smart contract will remind the responsible party of the specific consequences of failure to meet the requirements, and the shipper will also receive notification of a change in the status of the goods. The smart contract for real-time tracking of e-commerce logistics information is shown in Figure 11.

The network layer of blockchain is based on P2P network topology, with regulatory agencies (postal administration bureau), information service providers, and payment clearing institutions (commercial banks or third-party payment platforms) as the main nodes, which are connected to each other through the Internet. The blockchain technology protocol standards implemented by the state implement standardized definitions for the operation behavior and data specifications of each node. In addition, shippers and transporters can directly log in the data interface provided by the information service provider to conduct data exchange and transaction with the information service provider. The real-time tracking network of e-commerce logistics information is shown in Figure 12.

The operation mechanism of blockchain for real-time tracking of e-commerce logistics information is as follows. (1) The shipper will send the transportation demand to the information service provider, which will match the appropriate transportation provider for it. (2) After the shipper, information service provider, and transport provider reach an agreement, the transport provider and information service provider provide services and the shipper pays the freight, during which a large number of transaction data will be formed. (3) Logistics transaction data are converted into hash value to form block body, which is recorded to Merkle root and inserted into block head. (4) The block header already contains the random number (hash algorithm call required), the hash value of the previous block, and the timestamp. (5) The voting nodes on the alliance chain reach an agreement to transfer the newly generated logistics transaction blockchain to the previous block and then broadcast it to all nodes of the whole network. (6) All network nodes store the collected transaction data in their hosts for backup.

The logistics information tracing mechanism based on the alliance chain has the following characteristics: the logistics management department and the Ministry of transport are the two management nodes with supervision authority. It can solve the conflict between complete decentralization of blockchain and supervision and realize a certain degree of multi-centralization to change the drawbacks and disadvantages of centralized control. Information service providers are responsible for publishing information and maintaining the blockchain network on the blockchain. At the same time, the benefits of transaction fees can be obtained in the process of transaction completion and blockchain network operation. The real-time tracking alliance chain mechanism of e-commerce logistics information is shown in Figure 13.

## 6. Description and Hypothesis of Real-Time Tracking Model of E-Commerce Logistics Information Based on Blockchain Technology

In this article, the incentive mechanism contract model based on the constraint of information service providers is established under the asymmetric information about the effort level of the information service providers at the initial stage of the establishment of blockchain.

Assume that the carrier is on the data logistics traceability platform based on blockchain technology: *Q* represents the container, *a* carrier represents the carrier product, *e* represents the carrier's effort to operate transportation through the platform, and *m* (*m* > 0) represents the resources and news services satisfying the development of blockchain technology outputs. The value of *m* is positively correlated with the maturity. *ε* represents the external uncertainty factor, *g* represents effort cost coefficient, *π* is transport revenue of carriers, *h* represents the sum of utility brought to the information service providers by using the platform, *k* represents the unit subsidy provided by the information service providers, *ρ* represents the absolute risk avoidance measure of carriers, and the expected revenue formula of carriers can be obtained as follows:

(6) $$\begin{array}{c} E\pi =n\left(ae+m+\varepsilon \right)+bQk\left(a\right)-\frac{ge^{2}}{2}\text{.} \end{array}$$

When *a* = [0, 1], *n* = 0.5, *m* = 0.1, *g* = 5, *h* = 3, and *ρ* = 0.8, it is more conducive to the sustainable development of the carrier's own enterprise.

## 7. Summary and Prospect

To sum up, the changes of several parameters, such as the maturity of blockchain technology, the effort cost coefficient of transport operators, the absolute risk avoidance degree of enterprises, and the variance of uncertain factors, affect the incentive contracts provided by information service providers. It shows the theory, application and operation process of blockchain technology from three aspects of blockchain model architecture, blockchain technology architecture and operation mechanism, and systematically combs the decentralization of blockchain technology, which can solve the problem of information communication failure caused by the large number of participating nodes in the logistics industry, the trust problem caused by information asymmetry between nodes, and the centralized defect caused by the centralized data processing mode.

## Figures and Tables

**Figure 1:** Merkle root structure.

**Figure 2:** Operation architecture of e-commerce logistics.

**Figure 3:** Layered real-time tracking algorithm of logistics information in blockchain.

**Figure 4:** External operation system of blockchain logistics system.

**Figure 5:** External operation system of blockchain logistics system.

**Figure 6:** Structure of blockchain logistics management system.

**Figure 7:** E-commerce logistics transportation system.

**Figure 8:** Smart contract deployment and execution process.

**Figure 9:** Blockchain technology architecture for real-time tracking of e-commerce logistics information.

**Figure 10:** Blockchain structure of real-time tracking of e-commerce logistics information.

**Figure 11:** E-commerce logistics information real-time tracking smart contract.

**Figure 12:** E-commerce logistics information real-time tracking network.

**Figure 13:** Real-time tracking alliance chain mechanism of e-commerce logistics information.

**Table 1:** The information contained in the block.

Byte	Field	Content
5	Block size	Block size
82	Block head	Summary information
Uncertain	Block body	Trading content

**Table 2:** The advantages and disadvantages of blockchain classification.

Blockchain classification	Degree of decentralization	Advantage	Disadvantage
Private chain	Low	Protection of privacy	Low degree of decentralization
League chain	Middle	Operating under regulatory protection	High delay, power gathering, few nodes
Public chain	High	Completely decentralized	Low TPS, not suitable for large transactions

## Data Availability

The datasets used and analyzed during the current study are available from the corresponding author upon reasonable request.

## References

[1] Ma X., Li W., Wu J., Li W., Wu J. (2021). Research on the operation of e-commerce enterprises based on blockchain technology and bilateral platforms. *Wireless Communications and Mobile Computing*.

[2] Sharma K., Chaurasia B. K. Trust based location finding mechanism in VANET using DST.

[3] Chen C., Li D. (2021). Research on the detection and tracking algorithm of moving object in image based on computer vision technology. *Wireless Communications and Mobile Computing*.

[4] Su X., Liu Y., Choi C. (2020). A blockchain-based p2p transaction method and sensitive data encoding for e-commerce transactions. *IEEE Consumer Electronics Magazine*.

[5] Huang Y., Li X., Zhang G. (2021). The impact of technology perception and government support on e-commerce sales behavior of farmer cooperatives: evidence from liaoning province, China. *Sage Open*.

[6] Li Y., Zhang Y., Wang L., Guan X. (2020). Research on potential ground risk regions of aircraft crashes based on ads-b flight tracking data and gis. *Journal of Transportation Safety & Security*.

[7] Jayakumar J., Nagaraj B., Chacko S., Ajay P. (2021). Conceptual implementation of artificial intelligent based E-mobility controller in smart city environment. *Wireless Communications and Mobile Computing*.

[8] Li X., Huang D. (2020). Research on value integration mode of agricultural e-commerce industry chain based on internet of things and blockchain technology. *Wireless Communications and Mobile Computing*.

[9] Hongmei Z. (2021). A cross-border e-commerce approach based on blockchain technology. *Mobile Information Systems*.

[10] Cao K., Xu Y., Wu Q., Wang J., Liu C. (2021). Optimal channel and logistics service selection strategies in the e-commerce context. *Electronic Commerce Research and Applications*.

[11] Müller R. (2020). Proposal for an automated real-time vat collection mechanism in b2c ecommerce using blockchain technology. *International VAT Monitor*.

[12] Zhang H., Dong J. (2020). Prediction of repeat customers on e-commerce platform based on blockchain. *Wireless Communications and Mobile Computing*.

[13] Ghanbary H., Fathian M. (2021). Combination swot-ahp analysis for using blockchain in e-commerce. *Journal of Engineering and Applied Sciences*.

[14] Huang R., Yan P., Yang X. (2021). Knowledge map visualization of technology hotspots and development trends in China’s textile manufacturing industry. *IET Collaborative Intelligent Manufacturing*.

[15] Peng H., Yao Y., Zhu X., Zhou R., Zi X. (2022). Research on intelligent transportation and logistics tracking of long billet based on machine vision. *Journal of Electronic Imaging*.

[16] Li S. (2020). Structure optimization of e-commerce platform based on artificial intelligence and blockchain technology. *Wireless Communications and Mobile Computing*.

[17] Fan Y., Zhao L., Qin J. (2020). Research and verification on real-time interpolated timing algorithm based on waveform digitization. *IEEE Transactions on Nuclear Science*.

[18] Xu Z., Zhu G., Metawa N., Zhou Q. (2022). Machine learning based customer meta-combination brand equity analysis for marketing behavior evaluation. *Information Processing & Management*.

[19] Ding W., Wu L. (2021). Research on the selection of supply chain marketing models based on e-commerce service levels. *Proceedings of Business and Economic Studies*.

[20] Zuo J. (2021). Analysis of e-commerce characteristics based on edge algorithm and cox model. *Wireless Communications and Mobile Computing*.

[21] Susilo R. D., Daniawan B., Wijaya A., Suwitno (2021). The acceptance study of e-commerce customers based on tam. *Bit-Tech*.

[22] Liu J., Pan B., Zhang X., Li D. (2021). Mobile e-commerce information system based on industry cluster under edge computing. *Mobile Information Systems*.

[23] Zhang S., Fu L., Chen R., Mei Y. (2020). Optimizing the cargo location assignment of retail e-commerce based on an artificial fish swarm algorithm. *Mathematical Problems in Engineering*.

